# Deep Personal Multitask Prediction of Diabetes Complication with Attentive Interactions Predicting Diabetes Complications by Multitask-Learning

This article has been retracted.

**DOI:** 10.1155/2022/5129125

**Published:** 2022-04-20

**Authors:** Ming Zuo, Wei Zhang, Qi Xu, Dehua Chen

**Affiliations:** ^1^Glorious Sun School of Business and Management, Donghua University, Shanghai, China; ^2^School of Computer Science and Technology, Donghua University, Shanghai, China

## Abstract

**Objective:**

Diabetic complications have brought a tremendous burden for diabetic patients, but the problem of predicting diabetic complications is still unresolved. Our aim is to explore the relationship between hemoglobin A1C (HbA1c), insulin (INS), and glucose (GLU) and diabetic complications in combination with individual factors and to effectively predict multiple complications of diabetes.

**Methods:**

This was a real-world study. Data were collected from 40,913 participants with an average age of 48 years from the Department of Endocrinology of Ruijin Hospital in Shanghai. We proposed deep personal multitask prediction of diabetes complication with attentive interactions (DPMP-DC) to predict the five complication models of diabetes, including diabetic retinopathy, diabetic nephropathy, diabetic peripheral neuropathy, diabetic foot disease, and diabetic cardiovascular disease.

**Results:**

Our model has an accuracy rate of 88.01% for diabetic retinopathy, 89.58% for diabetic nephropathy, 85.77% for diabetic neuropathy, 80.56% for diabetic foot disease, and 82.48% for diabetic cardiovascular disease. The multitasking accuracy of multiple complications is 84.67%, and the missed diagnosis rate is 9.07%.

**Conclusion:**

We put forward the method of interactive integration with individual factors of patients for the first time in diabetic complications, which reflect the differences between individuals. Our multitask model using the hard sharing mechanism provides better prediction than prior single prediction models.

## 1. Introduction 

Diabetes [1] and its complications have been recognized as the most serious public health problem in the world. The global prevalence of diabetes among adults over 18 years of age increased from 4.7% in 1980 to 8.5% in 2014 [2]. Diabetic complications, including diabetic retinopathy, diabetic nephropathy, diabetic peripheral neuropathy, diabetic foot disease, and diabetic cardiovascular disease, contribute significantly toward life lost [3]. More than 50% of diabetes deaths resulted from cardiovascular and cerebrovascular complications, and 10% of those are from diabetic nephropathy [4]. Some scientific evidence has proved that diabetes complications can be avoided or delayed through diet, physical activity, medication, and regular screening and treatment [5]. For example, early detection and treatment of retinopathy that threatens vision can prevent or delay the occurrence of blindness and delay the development of diabetic nephropathy due to renal failure [6]. However, the management and control of diabetes are still poor in developing countries, especially in China. Many undiagnosed diabetic patients remain undiagnosed until diabetic complications occur. Hence, effective prediction of diabetes complications and treatment are key to saving patients' lives and improving their quality of life [1].

The discovery of diabetes risk factors and prediction of diabetic complications have been widely discussed in the scientific community [1]. Piri and his colleagues have used an integrated learning method to establish a diabetic retinopathy decision support system to solve the problem of low compliance of patients with diabetic retinopathy screening [7]. Other researchers also explored the possibility of using electronic records of patients to predict disease incidence [8, 9]. In view of the characteristics of people with type 1 diabetes, Marini has proposed a dynamic Bayesian network (DBN) [10] to predict the complications of patients with type 1 diabetes, especially those with diabetic nephropathy and cardiovascular disease [11]. However, so far, most of the research data have come from community residents or specific volunteers, which only contained limited information. Metabolic injury can be caused by protein glycation monitored by the level of hemoglobin A1C (HbA1c). HbA1c can effectively reflect the condition of the patient's blood glucose control in the past two months, and blood glucose is an index that directly measures the patient's present condition, whereas the insulin index is an important indicator to distinguish the type of diabetes of a patient. The aim of the present study is to use artificial intelligence [12] (AI) technology with multiple biochemical indicators to establish a predictive model for diabetic complications.

## 2. Materials and Methods

### 2.1. Data Collection and Clinical Evaluation

Data were derived from the patient data collected by the clinical diagnosis of diabetes in Ruijin Hospital of Shanghai, China. Each patient had a unique medical card number, and the diagnostic data of different departments were integrated according to the medical card number. There are three main monitoring indicators for diabetes. Among them, HbA1c can reflect the control level of blood glucose in the past two months; fasting insulin (INS) can effectively distinguish the type of diabetes; 2-hour postprandial blood glucose (2h PG) is an important standard to reflect the short-term condition of patients, and it is an indicator of the condition of hyperglycemic diabetic patients [13]. There are 8 treatment options for patients, including drugs, potassium chloride slow-release tablets, methazole tablets, and other treatment methods. Dosages are closely related to treatment options in nature, and different drugs can vary greatly. Doses of our drugs ranged from 10 mg to 500 mg. Among them, 10,847 patients with HbA1c were extracted with a total of 38,896 HbA1c, 9306 patients were extracted with fasting insulin, and 9166 patients were extracted with 2h PG. In addition to diabetes biochemical indicators, we also collected patients' blood pressure observations, treatment prescription, and the daily doses of medication.

### 2.2. Definitions and Diagnostic Criteria

HbA1c is determined by high-performance liquid chromatography (HPLC) [14], the normal value of which is 4%–6%. Blood glucose is a direct indicator of the patient's condition, and blood glucose between 7.78 and 11.1 m mol/L (140 to 200 mg/d L) within 2 hours postprandial indicates impaired glucose tolerance. Blood glucose at 2 hours postprandial >11.1 m mol/L (>200 mg/dL) was diagnosed as diabetes. Fasting insulin is an important index to distinguish the type of diabetes in patients. The normal reference value of fasting basal insulin for adults is 5–20 *μ*U/mL.

### 2.3. Statistical Analysis

The patient's blood pressure was divided into systolic and diastolic pressure, the former of which ranged from 100 to 192, with an average of 131.29, and the latter ranged from 46 to 249, with an average of 72.30. The incomplete data set will lead to many problems such as poor prediction effect, and we also adopt a series of methods to reduce this effect. The dataset is processed with null value processing, one-hot coding [15], normalization [16], sparse auto encoding, and prediction processing.

## 3. Methods

We used Acc (Accuracy), Precision, Recall, and F1 score to evaluate the experimental results. We used a long short-term memory [17, 18] sparse auto encoder (LSAE) to reduce the dimension and the interactive fusion method to compare the prediction effect of different models. It should be noted that we also compared multitasking separately. We compared the prediction results of interactive fusion and other multimodal fusion methods. Besides, we compared the experimental results of the LSAE with other dimensionality reduction models.

We set up comparative experiments according to five kinds of complications. Under the premise of considering only one complication, the five tasks in our deep personal multitask prediction of diabetes complication with attentive interactions (DPMP-DC) model could be transformed into five binary classification problems, which can be evaluated by the evaluation criteria of two classification problems. Through comparative experiments, we could conclude that our model has better performance than general bidirectional long short-term memory (Bi-LSTM) in classifying complications. In addition, we also compared with the classification prediction model of the Naive Bayesian model (NBM), support vector machine (SVM), convolutional neural network (CNN), and recurrent neural network (RNN).

## 4. Results and Discussion

We compared the experimental results of various models in different stages and discussed the experimental results. The average age of patients is 46 years. In terms of gender, the proportion of males is 35.64%, and that of females is 64.36%. The information of patients with diabetes complications is shown in Table 1. We take the diagnostic information table of a certain patient as an example for illustration. The input data format of the patient after data preprocessing is shown in Table 2. In the case of a patient, where the sex is male, a “10” is used, and a woman is represented by “01”; the age normalization is 0.5526; the systolic pressure is 0.619 after normalization; the diastolic blood pressure is 0.3646; the treatment plan is expressed in binary form, where “100” means the fifth treatment; the dose after normalization is indicated by the value of 0.5.

### 4.1. Comparison of Different Models for Predicting Five Diabetic Complications

In the prediction of diabetic retinopathy, the experimental results predicted by various models of diabetic retinopathy are shown in Table 3. We found that the accuracy of our model is 88.01% while that of the CNN was 75.90%. The accuracy of Bi-LSTM and DPMP-DC are more accurate than RNN and other models. However, in the prediction of patients with diabetic retinopathy, the recall rate of the DPMP-DC model was lower than that of other models, which indicated that in the multitask model, there were more errors in predicting patients although the overall accuracy was still accurate.

Table 4 shows the comparison results of various models of diabetic nephropathy. The prevalence rate of diabetic nephropathy data was high. 7352 out of 9166 patients had diabetic nephropathy. The accuracy of Bi-LSTM and DPMP-DC was similar. The model of predicting diabetic nephropathy presented the highest accuracy among the five complications. The accuracy of our model remained the highest, reaching 89.58%, which was much higher than that of the CNN and NBM. In terms of accuracy, our model was 0.73% higher than the Bi-LSTM model and 5.27% higher than the RNN. The performance of the DPMP-DC model was still better than that of all other baseline models in diabetic nephropathy.

Table 5 shows the comparison results of various models of diabetic peripheral neuropathy. In the prediction of complications of diabetic peripheral neuropathy, the accuracy of all models has been reduced. Among them, the overall evaluation index of the DPMP-DC model declined greatly because the correlation between various complications was strong. The CNN and Bi-LSTM have a good prediction effect on this complication, with an accuracy rate of 78.05% and 80.73%, respectively. Our model reached 86.77%, and other indicators of the prediction effect also performed best. The accuracy of our model was 5.03% higher than that of the best performing model in the baseline and 17.34% higher than the worst performance—SVM.

The experimental results of the prediction of various models of diabetic foot disease are shown in Table 6. The model of prediction diabetic foot disease has the least accuracy model of all complications. Although the accuracy of our model was only 80.56%, it is still much better than that of the models of the RNN (75.56%) and Bi-LSTM (72.11%). The NBM model was the worst, with an accuracy rate of only 65.34%. Our model could comprehensively consider other disease information, so the accuracy of the DPMP-DC model for diabetic foot disease was significantly higher than that of the two-way LSTM and other models.

The comparative experimental results of prediction of various models of diabetic cardiovascular disease are shown in Table 7. Our model had an accuracy rate of 82.48%, while the NBM, SVM, and CNN had a stable performance with an accuracy rate of about 70%. In comparison, the RNN had better prediction than other baseline models, with an accuracy rate of 78.40%. The accuracies of all prediction models for diabetic cardiovascular disease were low. The experimental results showed that DPMP-DC was better than the Bi-LSTM model and other models.

### 4.2. Comparison of RNN, LSTM, and Bi-LSTM in the Hidden Layer of Multitask Learning

Because the parameter setting in the model was more inclined to determine the direction of patients suffering from complications, the accuracy was low in the data set with fewer patients. However, such modification can ensure that the model had a better performance for the diseases with relatively average data. We used multitask prediction accuracy (MT-Acc) and missed diagnosis (Missdiag) as evaluation indicators for such a comparison process. Our comparative experimental results are shown in Table 8.

We used Bi-LSTM as the hidden layer method in multitask learning. We also used other models to replace the hidden layer model and carried out the experimental comparison. Taking diabetic foot as an example, our experimental results showed that the MT-Acc when using the RNN as a replacement model was 69.76% while that of Missdiag was 19.78%. The rate of Missdiag was much higher than that of the other two models. Using LSTM as the replacement model, the MT-Acc was 78.32%, while Missdiag was 11.25%. The MT-Acc of Bi-LSTM used in our model is 84.67%, while the rate of missed diagnosis was only 9.07%. The RNN ignored the information of long time series. The LSTM could not process the information before and after the sequence. The Bi-LSTM in our model had a better prediction effect and stability than the other two.

### 4.3. Comparison of Individual Interaction Fusion and Other Multimodal Fusion Methods

Our model interacted with individual factors and biochemical indicators of diabetes and was compared with the usual mode fusion method. The experimental results are shown in Table 9. We could further integrate the individual differences of patients as indicators of individual differences by combining the individual characteristics of patients. We compared and analyzed the prediction results of other multimodal fusion models under the condition that other processes remain unchanged. Our experimental results showed that the three models had the worst prediction effect in the way of “add” fusion. The MT-Acc of the RNN was 69.73%, and that of Bi-LSTM was 80.25%. Our DPMP-DC model uses three fusion methods to compare the prediction results. The experiment found that the effect of interaction fusion was the best, the MT-ACC was 84.67%, and the misdiagnosis rate was 10.15%.

## 5. Discussion and Analysis

We proposed a DPMP-DC model to process the data and effectively solved the problem of multitask prediction of diabetic complications. We used the LSTM with multitask learning (MTL-LSTM) model to predict multiple diabetes conditions. We used a way to interactively analyze diabetes biochemical indicators and individual factors and used the LSAE model to reduce dimensionality. In addition, on the premise of preserving sequence information, penalty terms can be added to obtain sequence features. This was an unprecedented attempt and progress in the field of diabetes complications. The greatest significance is that we proposed a new model that could effectively solve the prediction problem of diabetic complications and reflect individual differences.

Previous methods were mainly aimed at a single diabetic complication, and most of them mainly relied on the use of blood glucose indicator for prediction, ignoring other biochemical indicators, and the similarity of clinical characteristics in patient medical records. In addition, they were not suitable for predicting complications of diabetes.

The performance of our interactive fusion model was much better than that of other fusion methods. We thought that “Concat” and other fusion methods only used individual factors and biochemical indicators of patients. Our model took into account the individual differences of patients and made full use of these differences, combining with the biochemical indicators of patients, to achieve a more accurate prediction performance.

In diabetic foot disease and diabetic cardiovascular disease experiments, we could see that when using the DPMP-DC model, the data distribution was uneven and the prediction of the disease had better stability. This was also in line with the clinical expectations for the prediction model. In addition, our model also achieved good results in the other three complications. In addition, after cross-validation, our model had good stability, reflecting the advantages of multitask learning over single task prediction and other baseline models.

## 6. Conclusion

We introduce the original data set of diabetic patients. We preprocess the data, fill in the null data, and extract the sequence features. We mainly talk about the data divided into two parts. The first part is the biochemical indicators of diabetes and individual factors of patients. The other part is the types of complications that the patients suffer from. We use LSAE to extract feature sequences, interactive fusion to reflect individual differences of patients, and multitask learning to predict multiple complications, which yield good results. Different hospitals have different diagnostic methods, which may have different prediction effects. On the one hand, patients have multiple types of diabetes, and their constitutions are quite different. Our data are mainly for patients with type 2 diabetes. On the other hand, there are great differences in diagnoses, treatment programs, and monitoring indicators in different hospitals, such as imaging examination, drug administration plan, and dose. In order to further ensure that the model has better robustness, we will further verify the effect in the case of lack of cross-hospital data and clinical data. In the future, it is necessary to further add interpretable analysis to analyze the correlation between patient-monitoring indicators and complications so as to facilitate personalized prediction of patients' personal conditions and reflect individualized differences. In the supplementary material, we introduce the network structure of the model in detail. We use the DPMP-DC model to achieve the desired goal, but there are still some areas that can be improved in future clinical applications and deployments, which are shown as follows:

1. Due to the lack of data, niche detection indicators were not able to construct a reasonable predictive model. With a sound hospital database system, in-depth integration of artificial intelligence, and medical care, medical data sets will gradually realize more diabetes biochemical indicator support. It can enrich the learning ability and scope of the model and further improve the effect and universality of the prediction of complications.
2. If the clinical diagnosis data set of multiple hospitals can be combined, the diversity of the data set can be more effectively increased. The stability and practicality of the model can be tested, and the development and application of smart medicine can be promoted. We will further use some public data sets to verify the stability of the model and compare public data sets and clinical medical data.
3. In addition to the biochemical indicators of diabetic patients, combined with the diagnosis and monitoring data of diabetic drugs taken by the patients, it is currently possible to integrate the medication history of diabetic patients on the basis of achieving a more accurate prediction. We believe that in the future, combined with the diagnosis and treatment records of patients, we can further expand our model from the aspects of prevention and treatment of patients so that our model has better clinical application significance and value.

## Figures and Tables

**Table 1:** Characteristics of participants according to birth weight categories.

Monitoring indicators	Birth weight (grams)			
	Quantity	Min	Max	Mean
HbA1c^a^ (mmol/L)	38896	2.8	18.7	7.15
INS^b^ (*μ*U/ml)	29124	4.39	381	57.14
2h PG^c^ (mmol/L)	30646	0.41	121.42	11.59
Sex^d^ (female/male)	26334/14579	—	—	—
Age^e^ (years)	40913	21	95	66.51
SP^f^ (mmol/L)	386318	100	192	131.29
DP^g^ (mmol/L)	386318	46	249	72.30
Therapeutic method^h^	1048576	—	—	—
Dosage^i^	1048576	10.00	500.00	128.56

^a^HbA1c: HbA1c is a form of hemoglobin used to reflect the average plasma glucose concentration over a period of time (4–8 weeks); ^b^INS: insulin can regulate the metabolic process and promote the uptake and utilization of glucose by tissue cells. The normal value was 5–20 (*μ*U/ml); ^c^2h PG: blood glucose concentration 2 h after normal meal is less than 7.78 mmol/L (140 mg/dL); ^d^Sex: gender includes male and female; ^e^Age: it is the age of the patient; ^f^SP: systolic pressure, a systolic blood pressure of ≤130 mmHg (18.6 kPa) is called normal blood pressure; ^g^DP: diastolic blood pressure, the normal diastolic blood pressure in adults is 60∼90 mmHg (12 kPa); ^h^Therapeutic method: the treatment of diabetic patients, such as surgical treatment and intravenous injection; ^i^Dosage: represents the dose in the treatment regimen.

**Table 2:** Patient's individual factors and biochemical indicators after data processing results.

Medical card^a^	V3b397 ^∗∗∗∗∗∗^6457					
HbA1c	0.246	0.367	0.106	0.035	−0.099	−0.495
INS	−0.091	0.065	0.034	−0.374	−0.059	0.369
2h PG	0.235	0.134	0.586	−0.046	0.045	0.274
Sex^b^	1			0		
Age	0.5526					
SP	0.6197					
DP	0.3646					
Treatment^c^	100					
Dosage	0.5					

^a^Medical card: the patient's medical card number; ^b^Sex: “10” means male, and “01” means female: ^c^Therapeutic method: “100” means oral medication, and other frequencies are also encoded.

**Table 3:** Comparison of different models for predicting diabetic retinopathy.

Model	Evaluation index			
	Acc	Precision	Recall	F1
NBM^a^	68.43%	78.05%	75.44%	76.31%
SVM^b^	72.57%	76.64%	78.05%	72.06%
CNN^c^	75.90%	82.53%	80.58%	83.54%
RNN^d^	81.78%	84.36%	85.87%	82.10%
Bi-LSTM^e^	87.64%	87.74%	87.87%	87.81%
DPMP-DC	88.01%	88.46%	87.31%	87.88%

^a^NBM: naive Bayesian model; ^b^SVM: support vector machine; ^c^CNN: convolutional neural network; ^d^RNN: recurrent neural network; ^e^Bi-LSTM: bi-directional-long short-term memory.

**Table 4:** Comparison of different models for predicting diabetic nephropathy.

Model	Evaluation index			
	Acc	Precision	Recall	F1
NBM^a^	75.56%	76.64%	77.87%	80.01%
SVM^b^	80.78%	78.40%	77.87%	76.90%
CNN^c^	85.68%	80.58%	81.25%	81.10%
RNN^d^	84.31%	82.10%	84.56%	83.58%
Bi-LSTM^e^	88.85%	88.41%	89.23%	88.82%
DPMP-DC	89.58%	89.67%	89.77%	89.72%

^a^NBM: naive Bayesian model; ^b^SVM: support vector machine; ^c^CNN: convolutional neural network; ^d^RNN: recurrent neural network; ^e^Bi-LSTM: bi-directional-long short-term memory.

**Table 5:** Comparison of different models for predicting peripheral neuropathy.

Model	Evaluation index			
	Acc	Precision	Recall	F1
NBM^a^	71.58%	68.43%	72.31%	71.20%
SVM^b^	68.43%	72.38%	73.54%	72.47%
CNN^c^	78.05%	75.89%	77.78%	78.56%
RNN^d^	75.90%	77.78%	75.90%	75.00%
Bi-LSTM^e^	80.73%	80.23%	81.19%	80.71%
DPMP-DC	85.77%	84.72%	85.56%	85.14%

^a^NBM: naive Bayesian model; ^b^SVM: support vector machine; ^c^CNN: convolutional neural network; ^d^RNN: recurrent neural network; ^e^Bi-LSTM: bi-directional-long short-term memory.

**Table 6:** Comparison of different models for predicting diabetic foot disease.

Model	Evaluation index			
	Acc	Precision	Recall	F1
NBM^a^	65.34%	68.56%	66.59%	69.65%
SVM^b^	70.36%	70.31%	71.78%	72.10%
CNN^c^	72.11%	72.19%	74.66%	74.56%
RNN^d^	75.56%	73.54%	72.10%	73.18%
Bi-LSTM^e^	72.11%	71.46%	72.16%	71.76%
DPMP-DC	80.56%	79.82%	80.84%	80.33%

^a^NBM: naive Bayesian model; ^b^SVM: support vector machine; ^c^CNN: convolutional neural network; ^d^RNN: recurrent neural network; ^e^Bi-LSTM: bi-directional-long short-term memory.

**Table 7:** Comparison of different models for predicting diabetic cardiovascular disease.

Model	Evaluation index			
	Acc	Precision	Recall	F1
NBM^a^	70.36%	69.65%	72.38%	68.40%
SVM^b^	72.38%	71.46%	68.13%	66.56%
CNN^c^	71.46%	72.01%	71.46%	69.81%
RNN^d^	78.40%	74.38%	72.29%	72.10%
Bi-LSTM^e^	73.50%	74.38%	72.79%	73.58%
DPMP-DC	82.48%	83.05%	82.08%	82.56%

^a^NBM: naive Bayesian model; ^b^SVM: support vector machine; ^c^CNN: convolutional neural network; ^d^RNN: recurrent neural network; ^e^Bi-LSTM: bi-directional-long short-term memory.

**Table 8:** Comparison of RNN, LSTM, and Bi-LSTM results in hidden layer.

Model^a^	Evaluation index^b^	
	Accuracy	Missdiag
RNN	69.76%	19.78%
LSTM	80.32%	11.25%
Bi-LSTM	84.67%	9.07%

^a^Model: the model refers to the model selected in multitask learning, and the process remains consistent in other stages. The model is the result of replacing our model with the RNN and LSTM when the structure of other stages is unchanged; ^b^Evaluation index: according to the experimental results of multitask prediction, the model uses the evaluation indicators specified by us for comparison. The comparison here is different from the single task prediction in the previous part.

**Table 9:** Comparison of individual interaction fusion and other multimodal fusion methods.

Model	Concat^c^	Feature fusion			Evaluation index	
		Add^b^	Interaction^a^	Accuracy		Missdiag
RNN_Con^e^	√			70.38%		20.30%
RNN_Add^e^		√		69.73%		21.52%
RNN_Inter^e^			√	77.54%		18.15%
Bi-LSTM_Con^e^	√			74.76%		19.68%
Bi-LSTM_Add^e^		√		72.32%		23.10%
Bi-LSTM_Inter^e^			√	80.25%		16.50%
DPMP-DC_Con^e^	√			82.34%		13.76%
DPMP-DC_Add^e^		√		78.40%		15.10%
DPMP-DC			√	84.67%		9.07%

^a^Interaction: it stands for individual factors with attentive interactions; ^b^Add: “Add” is the constant number of channels and the addition of the feature map; ^c^Concat: it takes the number of channels increased, individual factors, and biochemical indicators as features and concatenates them as input data; ^e^*∗*_Con/Add/Inter: “*∗*” represents the base network used by the model, and it indicates which feature fusion method was used in the model.

## Data Availability

The diabetes data used to support the findings of this study are restricted by the Medical Ethics Committee of Ruijin Hospital, Shanghai Jiao-Tong University School of Medicine, in order to protect patient privacy. Data are available from Mingzuo, zm@rjh.com.cn, for researchers who meet the criteria for access to confidential data.

## Supplementary Materials

Supplementary Materials Figure 1: overall Architecture of the DPMP-DC model. Figure 2: LSAE was used to reduce the dimension of the input biochemical indicators. Figure 3: multitask LSTM learning for prediction. Figure 4: LSTM network structure. Figure 5: bi-LSTM frame structure.
